The article "Medical Image Captioning Using Optimized Deep Learning Model" was retracted in 2023. Reasons: signs of a paper mill; compromised peer review; unreliable results or conclusions.

# Medical Image Captioning Using Optimized Deep Learning Model

**DOI:** 10.1155/2022/9638438

**Published:** 2022-03-09

**Authors:** Arjun Singh, Jaya Krishna Raguru, Gaurav Prasad, Surbhi Chauhan, Pradeep Kumar Tiwari, Atef Zaguia, Mohammad Aman Ullah

**Affiliations:** ^1^Computer and Communication Engineering, Manipal University Jaipur, Jaipur, India; ^2^Manipal University Jaipur, Jaipur, India; ^3^Computer Science and Engineering, Jaipur Institute of Engineering and Management, Jaipur, India; ^4^Department of Computer Science, College of Computers and Information Technology, Taif University, P.O. Box 11099, Taif 21944, Saudi Arabia; ^5^Department of Computer Science and Engineering, International Islamic University, Chittagong, Bangladesh

## Abstract

Medical image captioning provides the visual information of medical images in the form of natural language. It requires an efficient approach to understand and evaluate the similarity between visual and textual elements and to generate a sequence of output words. A novel show, attend, and tell model (ATM) is implemented, which considers a visual attention approach using an encoder-decoder model. But the show, attend, and tell model is sensitive to its initial parameters. Therefore, a Strength Pareto Evolutionary Algorithm-II (SPEA-II) is utilized to optimize the initial parameters of the ATM. Finally, experiments are considered using the benchmark data sets and competitive medical image captioning techniques. Performance analysis shows that the SPEA-II-based ATM performs significantly better as compared to the existing models.

## 1. Introduction

Human beings have the potential to extract visual information from images [1–3]. The main objective is to utilize this human ability to generate meaning-full textual information from digital images to design automatic medical image captioning [4, 5]. Medical image captioning represents the content of an input image in a natural language by using various machine and deep learning models [6]. Thus, it initially extracts the content information and, afterward, it provides descriptive sentences [7, 8]. Recently, many recurrent neural network (RNN) and convolutional neural network (CNN) based medical image captioning models have been designed and implemented [9, 10].

Image captioning provides a variety of approaches that link the visual contents with normal language, e.g., explaining images with textual descriptions [11, 12]. In the existing literature, artificial neural network-based models were utilized to encode visual information with pre trained classification networks such as CNN and RNN [13]. The salient features of images were extracted for the efficient implementation of image captioning models [14–16].

The existing models have achieved significant results to obtain better captioning results from the images. However, the existing models do not consider the interplay between objects and stuffs [17, 18].

Recently, the encoder-decoder models have achieved significantly better results to efficiently extract the captions of medical images [19–21]. Initially, the features of the images are extracted using the CNN layers. The RNN model then utilizes the extracted features to extract shape-related information [22, 23]. LSTM is then utilized to obtain the textual information from the images. This process is then implemented again and again to extract end-level tokens [24–26]. Xiao et al. studied that encoder-decoder approaches are extensively utilized in medical image captioning, and the majority of them are implemented using single long short-term memory (LSTM) [27].

The main contributions of this work are as follows:

1. An efficient show, attend, and tell model is proposed. The show, attend, and tell model utilizes an encoder-decoder approach to generate the captions from medical images.
2. SPEA-II is used for the efficient selection of initial parameters of the proposed model.
3. Extensive experiments are considered by using the benchmark data sets and competitive medical image captioning models.

The remaining paper is structured as follows: section 2 presents the recent advancements in the field of medical image captioning.  Section 3 mathematically defines the SPEA-II-based ATM. Performance analysis is demonstrated in Section 4.  Section 5 provides the concluding remarks.

## 2. Related Work

Recently, many researchers have used deep learning and deep transfer learning models for the prediction and diagnosis of various kinds of patients [28–31]. Therefore, many medical image captioning models by considering deep learning and deep transfer learning have been proposed in the literature.

Zhang et al. proposed a visual aligning attention (VAA) model by using a novel visual aligning loss (VAL) function to build the model. VAL is computed by explicitly computing the feature correlation of attended image features and their respective word embedding vectors [32]. Oluwasanmi et al. designed a multimodal end-to-end Siamese difference captioning model (SDCM) to evaluate the potential information between two images. SDCM combines deep learning approaches with characteristics such as computing, aligning, and capturing, and disparity in images, to develop a corresponding language model probability distribution [33].

Xiao et al. implemented a deep hierarchical encoder-decoder network (DHN) for medical image captioning. DHN divides the functionalities of the encoder and decoder. It can evaluate the potential information by integrating the high-level semantics of language and vision to obtain medical captions [27]. Zakraoui et al. utilized natural language processing to evaluate the textual information in stories. Thereafter, a medical image captioning process using a pretrained deep learning approach is considered [34].

Wang et al. proposed a cascade semantic fusion (CSF) architecture to evaluate the potential characteristics to encode the content of medical images using an attention approach without considering the bells and whistles [35]. Yuan et al. designed an effective framework for captioning the remote sensing image. The framework is based on multilevel attention and multilabel attribute graph convolution [36].

From the related review, we can say that the development of an efficient image captioning model is still a challenging issue. Additionally, not much work is done to tune the initial parameters of medical image captioning models [37–41]. Therefore, using meta-heuristic techniques for initial parameter tuning issues (see [42, 43] for more details) is the main motivation behind this research work.

## 3. Proposed Methodology

In this paper, a novel show, attend, and tell model is implemented. A visual attention approach is introduced by considering the encoder-decoder approach. It has the ability to automatically concentrate on the salient objects of medical images to obtain descriptions in the decoder. The diagrammatic flow of the SPEA-II-based ATM is represented in Figure 1.

This model utilizes a convolutional neural network (CNN) as an encoder to obtain *L* vectors with *K* dimensions. Every vector represents a mask in the medical image. The convolutional layer's output is directly used to evaluate the feature vectors as

(1) $$\begin{array}{c} a=\left\{a_{1},\ldots ,a_{L}\right\},a_{i}\in {\mathbb{R}}^{K}. \end{array}$$

In the decoder part, LSTM is utilized for description generation. The feature vector in every iteration *t* is also considered to obtain the context vector as

(2) $$\begin{array}{c} z_{t}=\sum_{i=1}^{L}\alpha_{ti}a_{i}, \end{array}$$

where *z*_*t*_ defines the embodiment of the attention approach. *α*_*t*_ ∈ *ℝ*^*L*^ shows the attention weight vector of *t* iteration which follows ∑_*i*=1_^*L*^*α*_*ti*_=1. *a* can be approximated by using a neural network. A softmax activation function can be defined as

(3) $$\begin{array}{c} \alpha_{ti}\propto \;\exp\left\{f_{\mathrm{att}}\left(a_{i},m_{t-1}\right)\right\}. \end{array}$$

Thus, the proposed attention encoder-decoder model can be defined as

(4) $$\begin{array}{c} a=\text{Encoder}\left(I\right),\\ z_{t}=\sum_{i=1}^{L}\alpha_{ti}a_{i},\;\alpha_{ti}\in \mathbb{R},a_{i}\in {\mathbb{R}}^{K},\\ x_{t}=W_{e}S_{t},\;t\in \left\{0,\ldots ,N-1\right\},\\ p_{t+1}=\text{Decoder}\left(x_{t},z_{t}\right),\;t\in \left\{0,\ldots ,N-1\right\}. \end{array}$$

But SPEA-II-based ATM is sensitive to the initial parameters. Therefore, SPEA-II is utilized to optimize the initial attributes of SPEA-II-based ATM.  Figure 2 shows the flowchart of SPEA-II. For mathematical and other details of the SPEA-II and hyper-parameter tuning issues, see [44–46].

Initially, the random population is obtained using the normal distribution. Nondominated solutions are then computed and added to the Pareto set. Then, fitness is computed. Thereafter, selection, mutation, and crossover operators are used to generate new solutions. Again, the fitness of the computed solutions is computed. Finally, the nondominated solutions are again appended to Pareto set. These steps remain continuous till the termination criteria are not get satisfied.

## 4. Performance Analysis

The performance of the SPEA-II-based ATM is evaluated on the VQA-Med [47] medical image captioning dataset. To evaluate the effectiveness of the SPEA-II-based ATM, experiments are done in MATLAB 2013*a* on an Intel core processor with 16 − *GB* RAM. The remaining section discusses the visual and quantitative analysis of the SPEA-II-based ATM on medical images.

### 4.1. Visual Analysis

Figure 3 shows the visual analysis of SPEA-II-based ATM. It clearly shows that SPEA-II-based ATM is able to extract significantly remarkable information from the input medical images. It clearly shows that for Figure 3(a), the proposed model has presented a concise and accurate information as a Doppler ultrasound image. Similarly, for other figures, correct information is provided to the medical users, such as for Figure 3(b) axial plane, for Figure 3(c) nodular opacity on the left ≠ metastatic melanoma, and for Figure 3(d) skull and contents organ system. Also, if you see the number of generated words depends upon the information available in the image.

### 4.2. Quantitative Analysis

Figure 4 demonstrates the root mean square analysis of the SPEA-II-based ATM. It is observed that when the epoch is 7, the corresponding root mean square error = 0.78633. So, the values obtained from particles during epoch 7 are used as tuned parameters from SVM. It has been found that, at epoch 7, all the datasets, i.e., training, testing, and validation, are modelled toward root mean square error as 0. Therefore, SPEA-II-based ATM utilizes the optimal parameters to train the medical image captioning model.  Figure 5 represents the gradient, mean (mu), and validation tests of the SPEA-II-based ATM. It is found that till epoch 13, we have obtained gradient and mu as 1.4782 and 0.001, respectively, when validation tests are 6. Therefore, SPEA-II-based ATM has the ability to recognize captions with good performance. Also, mu as 0.001 shows that SPEA-II-based ATM does not suffer from the overfitting problem.

Figure 6 depicts the computed error bins of the proposed image captioning model when we have evaluated the difference between the actual and predicted classes. The difference is used to decompose the error into 20 different bins. It is found that, in the majority of the bins, the obtained error models are toward zero. The minimum error is evaluated at 9^th^ bin as −0.04836.

Figure 7 shows training, validation, testing, and the entire dataset, respectively, analyses. The SPEA-II-based ATM achieves remarkably good captions as the computed mean squared error (MSE) approaches toward 0.

Figure 8 represents the obtained confusion matrix of all seven (consider six core objects and others are represented by using the seventh class) classes of captions. It is observed that the majority of the computed classes lies in the true classes (i.e., in the diagonal matrix). Thus, SPEA-II-based ATM achieves better performance in terms of accuracy, F-score, sensitivity, specificity, etc. In Figure 8, class 0 is our true class, which means all other classes from 1 to 7 come under negative classes. Here, the value 34 at coordinate (0,0) indicates the true positive (*T*_*p*_) class, whereas the sum of all other diagonal classes shows the true negative (*T*_*n*_) class. Similarly, all vertical values represent corresponding false values. Therefore, in this figure, when we assume the target class as 0, we have false positive (*F*_*p*_)=2 and false negative (*F*_*n*_)=7.

Figures 9–13 demonstrate the performance analyses of SPEA-II-based ATM. In these figures, notched box-whisker boxplot analyses are evaluated. The interquartile range (IQR) is demonstrated using the boxes. The median of the evaluated data is shown using a red line. Notch shows a confidence interval near to the median value. If the notch size is smaller, then the given model obtains better results (i.e., with lesser variation) in every experiment.

Figure 9 illustrates the comparative analyses among the existing medical image captioning models and the SPEA-II-based ATM in terms of accuracy. It demonstrates that the SPEA-II-based ATM achieves significant accuracy values than the competitive medical image captioning models. The SPEA-II-based ATM achieves an average accuracy as 1.234% over the competitive medical image captioning models.

Figure 10 shows the f-measure analysis of the SPEA-II-based ATM. In terms of f-measure, SPEA-II-based ATM achieves a mean improvement as 1.178% over the competitive models [48].

Figure 11 demonstrates the specificity analysis of the SPEA-II-based ATM. It SPEA-II-based ATM shows an average improvement as 1.319% over the competitive medical image captioning models.

Figure 12 shows the sensitivity analysis of the SPEA-II-based ATM. It is evaluated that the SPEA-II-based ATM shows an average improvement as 0.983% over the competitive models. Therefore, the SPEA-II-based ATM provides significant details about the medical images.

The kappa statistics analysis is shown in Figure 13. It is found that the SPEA-II-based ATM obtains better kappa values than the existing models. The average enhancement in terms of kappa statistics is found to be 0.9382.

## 5. Conclusion

Medical image captioning provides the visual information of medical images in the form of natural language. In this paper, a novel show, attend, and tell model has been designed and implemented. A visual attention mechanism based on the encoder-decoder structure has been introduced. However, SPEA-II-based ATM suffers from hyperparameter tuning issues. Therefore, in this paper, SPEA-II has been used to tune the initial attributes of an SPEA-II-based ATM. Finally, experiments have been considered using the benchmark data sets and competitive medical image captioning models. Extensive experiments demonstrated that SPEA-II-based ATM outperforms the existing medical image captioning models. In this paper, only SPEA-II is used to tune the parameters of the proposed model. Therefore, in the near future, an efficient metaheuristic technique will be proposed to achieve better results. Additionally, the proposed model can be extended for other kinds of outdoor images.

## Figures and Tables

**Figure 1:** Proposed deep learning based medical image captioning.

**Figure 2:** Flowchart of strength Pareto evolutionary algorithm-II (SPEA-II).

**Figure 3:** Proposed deep learning based medical image captioning. (a) Doppler ultrasound scan. (b) Axial plane. (c) Nodular opacity on the left ≠ metastatic melanoma. (d) Skull and contents organ system.

**Figure 4:** Performance analysis of SPEA-II-based ATM.

**Figure 5:** Mean, gradient, and performance check analysis of SPEA-II-based ATM.

**Figure 6:** Error histogram of SPEA-II-based ATM with 20 bins.

**Figure 7:** Performance analysis of error plots on medical image captioning dataset.

**Figure 8:** Confusion matrix analysis of the medical image captioning dataset.

**Figure 9:** Performance analysis of SPEA-II-based ATM for medical image captioning in terms of accuracy.

**Figure 10:** Performance analysis of the SPEA-II-based ATM model for medical image captioning in terms of F-measure.

**Figure 11:** Performance analysis of the SPEA-II-based ATM model for medical image captioning in terms of specificity.

**Figure 12:** Performance analysis of the SPEA-II-based ATM model for medical image captioning in terms of sensitivity.

**Figure 13:** Performance analysis of the SPEA-II-based ATM model for medical image captioning in terms of kappa statistics.

## Data Availability

The data used to support the findings of this study are freely available at https://cvit.iiit.ac.in/usodi/Docfig.php.
